# Deep Learning in Ischemic Stroke Imaging Analysis: A Comprehensive Review

**DOI:** 10.1155/2022/2456550

**Published:** 2022-11-14

**Authors:** Liyuan Cui, Zhiyuan Fan, Yingjian Yang, Rui Liu, Dajiang Wang, Yingying Feng, Jiahui Lu, Yifeng Fan

**Affiliations:** ^1^School of Medical Imaging, Hangzhou Medical College, Hangzhou, Zhejiang, China; ^2^Centre of Intelligent Medical Technology and Equipment, Binjiang Institute of Zhejiang University, Hangzhou, Zhejiang, China; ^3^School of Medicine and Biological Information Engineering, Northeastern University, Shenyang, China

## Abstract

Ischemic stroke is a cerebrovascular disease with a high morbidity and mortality rate, which poses a serious challenge to human health and life. Meanwhile, the management of ischemic stroke remains highly dependent on manual visual analysis of noncontrast computed tomography (CT) or magnetic resonance imaging (MRI). However, artifacts and noise of the equipment as well as the radiologist experience play a significant role on diagnostic accuracy. To overcome these defects, the number of computer-aided diagnostic (CAD) methods for ischemic stroke is increasing substantially during the past decade. Particularly, deep learning models with massive data learning capabilities are recognized as powerful auxiliary tools for the acute intervention and guiding prognosis of ischemic stroke. To select appropriate interventions, facilitate clinical practice, and improve the clinical outcomes of patients, this review firstly surveys the current state-of-the-art deep learning technology. Then, we summarized the major applications in acute ischemic stroke imaging, particularly in exploring the potential function of stroke diagnosis and multimodal prognostication. Finally, we sketched out the current problems and prospects.

## 1. Introduction

Stroke is recognized as an acute cerebrovascular disease, leading to the second main factor of disability and death worldwide, which resulted in a global substantial financial burden (approximately 34 billion dollars per year) [1, 2]. Stroke can be divided into ischemic stroke (which accounted for more than 87% of all stroke patients) and hemorrhagic stroke [3]. The time window for treating stroke disease treatment in the acute phase is generally 6 hours after onset. Therefore, it requires rapid decisions and appropriate interventions from clinicians [2, 3]. Neuroimaging techniques (including CT and MRI) have become an integral approach to acute stroke detection, characterization, and prognosis [4]. However, it is a great challenge for neuroradiologists due to its similar intensity and shape to stroke lesions produced by artifacts in CT or MRI [5, 6]. As a new computer-aided diagnostic method, artificial intelligence (especially deep learning) might provide a novel approach to overcoming these obstacles [7]. It enables end-to-end learning and offers more precise medical treatment and reasonable clinical decisions, including triage, quantification, surveillance, and prediction of disease [5]. This review is aimed at summarizing the current status of deep learning-driven acute ischemic stroke applications and analyzing the role of deep learning on rapid stroke lesion identification, accurate diagnoses, and timely therapy.

Over the past decades, various machine learning techniques, including logistic regression (LR) [8], linear discriminant analysis (LDA) [9], support vector machines (SVM) [10], decision trees (DT) [11], random forests (RF) [12], and neural networks [13], have been applied. These approaches rely largely on predefined engineered features, such as the shape, the texture, and the distribution of pixel intensities (histogram) obtained from computer programs. Then, these features, identifying potential imaging-based biomarkers for clinical decision-making support, are utilized as inputs to innovative machine learning models [14]. SVM improved the identification of carotid atherosclerosis (CA) from magnetic resonance brain images and prevented ischemic stroke patients with an ACC of 97.5% [15]. The combination of RF methods with geodesic active contour (GAC) technology can automatically segment cerebrospinal fluid (CSF) in CT images for early cerebral edema identification, a major medical complication after ischemic stroke [16]. The LR method for CT angiography (CTA) lesion analysis and differentiation of floating intraluminal thrombus and atherosclerotic plaque is helpful for the selection of stroke treatment plan, and the sensitivity of this method reaches 87.5% [17]. Predicting the presence and laterality of a perfusion deficit on CT perfusion scans using ANN can promote further therapy. ACC reached 85.8% in CT perfusion images of 396 patients [18]. ML approaches were employed on various datasets for solving various stroke problems for a better healthcare system and further investigation [19]. However, conventional machine learning mainly uses feature engineering, requiring manual extraction and data cleaning. Problems such as optimizing image features and being susceptible to multimodal image interference need to be further explored and improved [20].

Deep learning is a subset of machine learning and an innovative application of artificial intelligence (AI), owning partly to its algorithm characteristics that automatically capture the hierarchical and complex features from raw input data [21–23]. Multilayer deep neural networks exert a positive function on huge challenging task solutions through mimicking the perception of the human brain and transforming “low level” into “high level,” especially in imaging classification, natural language process, or bioinformatics [24, 25]. Recently, the medical image process has developed into a hot research field of deep learning, involving multiple tasks of disease classification [26], lesion localization and segmentation, and imaging reconstruction [27]. As a consequence, deep learning has been widely applied to the diagnosis and management of stroke, for instance, the prediction of clinical outcomes of AIS patients [28]. In contrast to conventional machine learning methods, deep CNN learning is not relying on hand-crafted features. Complex features from data are extracted and expressed automatically by DL when locating the stroke lesion core in CT or MRI [29]. Deep learning not only saves time and effort but also captures the pixel-level information of the lesion, which is beneficial to improve the accuracy of diagnosis and prognosis [30]. As shown in Figure 1, the analysis of many typical deep learning models and applications of deep learning in ischemic stroke imaging is presented.

The rest of this paper is organized as follows. In Section 2, we exhibit the historical development of deep learning, including convolutional neural network (CNN), recurrent neural network (RNN), autoencoder (AE), restricted Boltzmann machine (RBM), transformer, and transfer learning (TL).  Section 3 discusses the applications of deep learning to stroke management in five main areas. Finally, we present outlook in Section 4.

## 2. Deep Learning Models

Deep learning (DL), derived from artificial neural networks (ANNs), mimics human brain intelligence in increasingly sophisticated and independent ways [31]. In 1989, LeCun et al. originally applied the CNN model for image recognition of handwritten characters, consisting of four parts (a convolutional layer, a pooling layer, an activation function, and a fully connected layer) [32]. In 2012, AlexNet won the championship in the ImageNet competition far surpassed second place, and since then, CNN has developed promptly along with the emergence of many typical CNN architectures [33], for example, VGGNet [34], GoogLeNet [35], and ResNet [36]. At present, CNN has become a relatively extensive network structure in medical imaging [37].

Recurrent neural network (RNN) is a special memory-based deep neural network, which is different from CNN, not only considering the network's input at the previous moment but also memorizing it for transmission to the next moment [38]. Considering chronological tasks, the RNN application is more extensive. To solve the gradient explosion or disappearance problem when RNN is backpropagated, long short-term memory (LSTM) was proposed [39]. The core of LSTM is adding three important gating units to the recurrent layer, including the input gate, forget gate, and output gate. Choi et al. [40] invented CNN-Bidirectional LSTM to predict stroke on raw EEG data, with an accuracy of 0.94. Additionally, Do et al. developed a recurrent residual convolutional neural network (RRCNN) combined with VGG16 and ResNet for the binary classification of Alberta Stroke Program Early Computed Tomographic Score (ASPECTS) using DWI in acute ischemic stroke patients, with an accuracy of 87.3% and AUC of 0.941 [41].

Autoencoder, a typical unsupervised deep learning model, is separated into encoding and decoding parts (encoder and decoder) [42]. The former can learn the hidden features of the input data, while the latter can reconstruct the original input data with the learned new features. Common applications of autoencoder contain image denoising and dimensionality reduction [30], for instance, denoising autoencoder (DAE) [43], sparse autoencoder (SAE) [44], variational autoencoder (VAE) [45], and contractive autoencoder (CAE) [46]. In ischemic stroke lesion analysis, Praveen et al. proposed a stacked sparse autoencoder (SSAE) architecture for accurate segmentation of ischemic lesions from MR images and performed perfectly on the publicly available Ischemic Stroke Lesion Segmentation (ISLES) 2015 dataset, with an average precision of 0.968, average Dice coefficient (DC) of 0.943, and the accuracy of 0.904 [47].

Restricted Boltzmann machine (RBM) is a random generative neural network that learns probability distributions from input datasets. The connections between neurons are bidirectional and symmetrical presented in Figure 2(d). This means that information flows in both directions during training and use of the network and that the weights are the same with the information. It can be used for dimensionality reduction, feature extraction, and collaborative filtering [48]. The RBM neurons are all binarized; that is to say, there are only two states, including activation and inactivation (0 and 1). In ischemic stroke lesion analysis, Pinto et al. used RBM to extract features from lesions and blood flow information from different MRI images to predict the final stroke lesion. On the publicly available ISLES 2017 test dataset, they evaluated their model and achieved a Dice score of 0.38, a Hausdorff distance of 29.21 mm, and a mean symmetric surface distance of 5.52 mm [49].

The transformer predisposed by Google provides a parallelized way of processing sequential data based on the attention mechanism (AM), which is much faster than CNN and RNN structures and very good at handling long-term dependencies [50]. Therefore, transformers have become the innovative deep learning model. As shown in Figure 2(e), the model mainly consists of multiple encoders and multiple decoder layers superimposed. Recently, transformers have accomplished impressive results in medical image segmentation tasks [51]. Based on the U-Net structure, Cao et al. progressed the SWIN-Unit transformer algorithm, superior to U-Net and other models in multiorgan and heart segmentation tasks, with a DSC value of 0.9 [52]. In ischemic stroke lesion analysis, the model, including CNN and transformer for encoding and the multihead cross-attention (MHCA) module for decoding, leads to stroke lesion morphology and edges with a Dice of 73.58% [53]. Transformers can be introduced to process data with different scanner models or multimodal data. Tang et al. proposed a novel unsupervised approach to fuse multimodal medical images via a multiscale adaptive transformer termed MATR and extended the method to address other biomedical image fusion issues, obtaining satisfying fusion results and generalization capability [54]. Karimi et al. proposed a convolution-free transformer network architecture that outperforms FCN-like architecture in both the task of segmenting multimodal 3D medical images (T2 MRI and MRI) and the task of pretrained networks augmented with unlabeled images [55]. Jiang et al. proposed SwinBTS, a new 3D medical picture segmentation approach, which combines a transformer, CNN, and encoder-decoder structure to define the 3D brain tumor semantic segmentation job and achieves excellent segmentation results on the public multimodal brain Tumor datasets of 2019-2021 (include T1,T1-ce,T2,T2-Flair) [56]. A novel network O-Net combining CNN and transformer for segmentation and classification of medical images was proposed by Wang et al. On the synaptic multiorgan CT dataset and the ISIC 2017 challenge dataset, the model realizes competitive performance and good generalization ability [57].

Transfer learning (TL) is a popular method of deep learning that is widely used in medicine [58]. The principle of the method is to reapply a pretrained model to another task. Transfer learning offers a suitable framework to take previously learned correlated knowledge and applies it to solve a new problem, particularly suitable for small data issue [59]. For example, to predict the risk degree of developing stroke disease with patient history (e.g., hypertension and diabetes mellitus), Chen et al. designed a multi-input hybrid transfer learning network structure. In addition, this method could overcome the limitations of label imbalance [60]. Zhang et al. proposed an intradomain task-adaptive transfer learning method to predict the time after stroke onset (TSS) in patients. The results showed a predictive AUC of 0.74 for TSS less than 4.5 h, indicating potential therapeutic implications for patients with unknown TSS [61].

## 3. Clinical Applications of Deep Learning in AIS

### 3.1. Early Stroke Diagnosis/Time from Onset

Stroke management highly depends on the NCCT and MR images. Inclusion criteria for acute ischemic stroke are as follows: first, patients with suspected ischemic stroke should undergo an NCCT scan to exclude the intracranial hemorrhage possibility [62]. Due to the low sensitivity of NCCT for hyperacute AIS, the sensitivity for hemorrhage is very high. Meanwhile, within the 90-minute time window after the onset of middle cerebral artery (MCA) occlusion, both the high-density MCA sign and the Sylvian MCA point sign are obvious signs of NCCT and are among the earliest visible signs of ischemia [63]. MRI can identify abnormal lesions in the acute stage of ischemic stroke [64]. DWI is gradually being recognized as the gold standard for the diagnosis of acute ischemic stroke, with a sensitivity of 73%-92% for hyperacute ischemic stroke detection within 3 hours of onset, and it detects deficiency beyond 6 hours after onset [48]. The sensitivity of hemorrhagic stroke had already reached 100%, while DWI combined with PWI can increase the diagnostic sensitivity of acute ischemic stroke (about 97.5%) and provide physiological information such as ischemic penumbra [65].

Especially, multiple studies have reported the potential of deep learning systems for the rapid and automated diagnosis and identification of ischemic stroke. The AI-based approach can exert synthesized function on clinical data, including clinical symptoms, medical history, family history, and neuroimaging features [66]. Deep learning has been extensively applied for early stroke diagnosis analysis (Table 1). Litjens et al. exhibited a 3D CNN and extracted contralateral features and anatomical atlas information to identify MCA, achieving an AUC of 0.996 and a precision-recall AUC of 0.563 in a voxel-level evaluation. Although the results are not yet at a level for routine clinical use, they are still encouraging [67]. It is exciting to see Lisowska et al. making further progress; they developed a deep convolutional neural network (DCNN) model to identify hyperdense middle cerebral artery sign (HMCAS) on CT, and the results proved that the model was compared with the diagnostic performance of neuroradiologists with the AUC of 0.869 [68]. Furthermore, Shinohara et al. developed an ANN model to identify and differentiate acute cerebral ischemia (ACI) and stroke mimics from patients within 4.5 hours of symptom onset. This method got great performance for the ACI diagnosis and differentiate ACI from SM cases with a precision of 92% [69]; however, this method presented limited generality. Researchers also proposed a deep symmetric 3D convolutional neural network (DeepSym-3D-CNN) based on the symmetry property of the human brain to learn diffusion-weighted imaging (DWI) and apparent diffusion coefficient (ADC) difference features for automatic diagnosis of ischemic stroke disease with an AUC of 0.850 [70]. This deep learning method is novel that exploited the symmetry of the human brain, but with a small amount of DWI data. As discussed above, future studies exploring stroke diagnosis on thin-section CT or MR could provide the DL algorithm with more valid features of the lesion and contribute to improving the sensitivity of the AI for automatic diagnosis. In addition, external validation should be enhanced by using more external data to validate the generalization capabilities of the models.

### 3.2. Automated ASPECTS Calculation

In the early time window after stroke onset (i.e., within 6 hours), it is difficult to discern the boundaries of the lesion on CT, particularly in white matter where the signal-to-noise ratio is poor. Therefore, a semiquantitative approach such as Alberta Stroke Program Early Computed Tomography Score (ASPECTS) is necessary for assessing the extent of infarct-related alterations in a rapid and reproducible fashion in MCA ischemic stroke patients [71]. The ASPECTS plays an important role in the early prediction of infarct core for middle cerebral artery (MCA) territory ischemic strokes and the suitability for reperfusion therapy [72]. It assesses 10 regions (Figure 3) within the MCA territory for early signs of ischemia, and the result score ranges from 0 to 10, where 0 indicates ischemic involvement in all 10 regions, while 10 indicates no early signs of ischemia. The guideline of AHA/ASA (American Heart Association/American Stroke Association) has incorporated ASPECTS ≥ 6 in their recommendations for the selection of patients for endovascular thrombectomy [73]. Hence, the score is currently a key component in evaluating the appropriateness of receiving endovascular thrombectomy. Unfortunately, the assessment of ASPECTS is more dependent on the experience of the radiologist.

Several AI software offerings which perform automated ASPECTS evaluation have been assessed in clinical settings. It helps physicians diagnose ischemia and offer a more consistent interpretation. Until now, two of them using machine learning algorithms are commercially available, for example, e-ASPECTS software (Brainomix, Oxford, UK) and RAPID-ASPECTS (Siemens Healthcare GmbH, USA) [74]. Studies have displayed the feasibility of software such as e-ASPECT and RAPID-ASPECTS to assess CT images. In recent years, the software has achieved a similar or even better diagnosis than radiologists. Nagel et al. compared RAPID-ASPECTS and e-ASPECTS to 2 experienced radiologists, finding that e-ASPECTS exhibited a better correlation with expert consensus [75]. Goebel et al. compared 3 neuroradiologists with e-ASPECTS, finding that the neuroradiologists had a better correlation with infarct core that was judged on subsequent imaging than the software [76]. Guberina et al. compared RAPID-ASPECTS (iSchemaView) to 2 neuroradiologists, finding that the software showed a higher correlation with expert consensus than each neuroradiologist [77]. However, traditional machine learning-based algorithms are limited because appropriate discriminating features must be defined by human developers and require to be manually extracted. Recently, end-to-end deep learning-based algorithms have presented a promising performance in medical image analysis tasks [78]. Deep learning has been extensively used for automated ASPECTS calculation (Table 2).

In 2021, Naganuma et al. conducted a study on automatic ASPECTS calculation of ischemic stroke using noncontrast computed tomography (CT). In this study, they compared a deep learning-based algorithm (3D-BHCA) to 5 stroke neurologists, finding that the region-based and score-based analyses of 3D-BHCA model were superior or equal to those of stroke neurologists overall [79]. This study has achieved good classification outcomes than conventional approaches. However, the study lacks external validation and reperfusion effect studies, as well as patients with old cerebral infarction and cerebral hemorrhage, which may interfere with the classification outcomes of the model.

DWI-ASPECTS is derived from CT-ASPECTS as a tool to semiquantify early ischemic alterations [41, 80, 81]. Innovatively, using diffusion-weighted imaging (DWI), Do et al. developed recurrent residual convolutional neural network (RRCNN) algorithm for the automatic binary classification of the ASPECTS in acute stroke patients with an AUC of 94.1%, indicating that the performance is better than 3DCNN. However, this study presents a global estimation of DWI-ASPECTS rather than a classification of individual DWI-ASPECTS regions [41]. Cheng et al. developed a deep learning-based automatic software tool (eDWI-ASPECTS) which was equivalent to the diagnostic efficiency of senior neuroradiologists in the evaluation of 10 individual ASPECTS regions, although there are uncertainties in the scoring rules of DWI-ASPECTS. Compared to CT, the initial description of the score is not yet clear [81]. In conclusion, the criteria for DWI-ASPECTS evaluation will be necessary for the future.

### 3.3. Detection of Large Vessel Occlusion

Most cases of ischemic stroke are caused by acute intracranial arterial thromboembolism. Currently, intravenous tissue plasminogen activator (IV-tPA) combined with endovascular thrombectomy (EVT) is the standard therapeutic scheme for patients with AIS induced by large vessel occlusion (LVO) [82]. Although LVO accounts for up to 38% of AIS, it is responsible for 60% of stroke-related disabilities and 90% of stroke-related deaths [83]. EVT has been demonstrated to considerably improve prognosis within 6 h from symptom onset [84, 85]; however, only 27% of patients who are eligible for thrombectomy receive EVT. Additionally, each of delayed 30 min in EVT decreases favorable outcomes by 11% [86]. Thus, systems for automatical and prompt detection of LVO have the potential to improve the rates of EVT and promote the chance of receiving appropriate reperfusion therapy in AIS patients, thereby contributing to neurological recovery.

The most critical application of CT angiography (CTA) is to detect large vessel occlusions (LVO). Several documents involving the Automated Large Arterial Occlusion Detection in Stroke Imaging (ALADIN) trial have been published by using AI algorithms with CTA datasets for identifying LVO (Table 3). For example, Amukotuwa et al. used Rapid CTA to detect intracranial anterior circulation LVOs with high diagnostic sensitivity (0.94) and NPV (0.98), as well as moderately high specificity (0.76) [87]. Furthermore, a CNN has been reported to be possibly used for detection of the head and neck CTAs, which indicates an 82% sensitivity and 94% specificity in a study with 650 persons. In practice, this can offer the possibility of early alerting a senior physician to help with task prioritization [88]. Shaham and R L R proposed a DeepSymNet model for automatic detection of ischemic stroke lesion areas in CTA, inspired by the Siamese network, with AUC 0.914 (CI0.88-0.95) and AUC 0.899 (CI 0.86-0.94) for original cerebral CTA volumes and brain tissue images, respectively [89]. The network is sensitive to symmetric alterations in blood vessels and brain structures, which can detect AIS lesions by effectively learning the contralateral lesion-free cerebral hemisphere from CTA images [90]. Yu et al. firstly established a three-tier diagnostic tool using machine learning and deep learning that was based on the structured clinical data with nonstructured NCCT imaging data for LVO diagnosis, which achieved superior performance with the AUC of 0.847, potentially improving the prehospital triage systems for AIS [91]. Nevertheless, the NCCT brain scans are thick-cut, and lacking prospective validation and angiogram within the acute setting is the main shortcoming of this study.

Multiple commercial software platforms are available for the automatic detection of LVO on CTA, such as Brainomix e-CTA (Brainomix Ltd.), Rapid CTA, Rapid LVO (iSchemaView), and Viz LVO (Viz.ai, California, USA). Brainomix e-CTA and Viz LVO utilize CNNs to analyze CTAs for LVO detection, while Rapid LVO indirectly detects LVO based on the asymmetry of CTA collateral blood vessel density [5]. These software tools also analyze CT/MRI perfusion, generating perfusion maps to estimate the stroke core and penumbra. In 2021, McLouth et al. validated a commercially available deep learning-based tool that performed well in the LVO cohort, with an accuracy of 98.1% [92]. Despite these technological innovations, there is still a dearth of studies involving rigorous comparison or validation for LVO detection tools. Thus, it is necessary to detect LVO by combining angiogram with thin-cut scans, as well as establish prospective validation in the future.

### 3.4. Utilizing Deep Learning for Evaluation of Ischemic Core and Penumbra/Prognosis

The volumes in the ischemic core (irreversibly damaged tissue) and penumbra (potentially salvageable ischemic tissue) are of great significance for the outcomes in AIS patients. However, the manual segmentation of the ischemic core and penumbra is a time-consuming and laborious mission, with inconsistency across raters [64]. Both the ischemic core and the penumbra area are irregular in shape due to the time from symptom onset, vessel occlusion site, and collateral status. There is a lot of noise related to lesion signals, such as leukoaraiosis and T2 shine-through effects; besides, tissue defects may further hamper lesion segmentation [93]. Therefore, it is challenging for radiologists to manually annotate the lesion area at the pixel level.

For clinical diagnosis and treatment, MRI and CTP are usually used to evaluate the ischemic core and penumbra. Compared to CT, magnetic resonance imaging (MRI) with diffusion-weighted imaging (DWI) sequence is much more sensitive for early ischemia detection [94]. Threshold-based approaches are widely used internationally to determine ischemic core with apparent diffusion coefficient (ADC) < 600 × 10^−6^ mm^2^/s and penumbra regions with specific time to maximum (Tmax) ≥ 6 s. The perfusion parameters have been outlined in the DEFUSE III trial [95], defining inclusion criteria as core volume < 70 mL, mismatch ratio (MMR) > 1.8, and mismatch volume (MM Vol) > 15 mL.

Several kinds of commercial software mainly use segmentation threshold to predict core infarct area and ischemic penumbra, for example, Rapid, F-stroke, E-stroke, and Vitra [96]. However, Koopman et al. have noted that CTP maps are unreliable in about 13% of cases when using Rapid, and most maps are not reliable for patients with erroneous Tmax calculations, some cases showing bihemispheric penumbra. The comparative analysis of these software results in significant differences in calculation outcomes due to different basic algorithms [97]. Furthermore, these threshold-based approaches fail to capture the complexity of infarct evolution in stroke. Currently, decision-making in acute ischemic stroke is mainly based on the time domain, which does not take into account the biological differences among patients.

The approach based on deep learning can automatically extract the lesion features at the pixel level and then classify and segment them. It has become a potential technique for segmenting core infarct and penumbra at home and abroad. Of course, it is an increasingly important part of decision support and shows some promising results. Deep learning has been applied to many aspects of the ischemic core and penumbra, and the literature is summarized in Table 4. Chen et al. utilized CNNs composed of MUSCLE Net and EDD Net in a study of segmenting stroke lesions automatically in 741 subjects by DWI, and the performance is comparable to manual segmentation [98]. Ho et al. developed an autoencoder structure model, which could extract high-dimensional imaging features from PWI image data, and used machine learning classifiers to locate stroke regions, achieving an AUC of 0.68, which is 10% better than the current traditional clinical method with AUC of 0.58 [99]. Sheth et al. designed a deep symmetry-sensitive convolutional neural network (DeepSymNet) based on the maximum likelihood method to evaluate the volume of large vessel occlusion with AUC of 0.88 and determined infarct core as defined by CTP-RAPID from the CTA with AUC of 0.88 and 0.90 (ischemic core ≤ 30 mL and ≤50 mL). The advantage of this method is that it does not require any prior knowledge, which greatly reduces data workload preprocessing in the early stage [100].Öman et al. detected AIS using 3D-CNN from CTA source images of 60 patients. This is the first study applying 3D CNN to CTA source images for ischemic stroke detection and achieving high sensitivity and specificity [101].

More recently, Nielsen et al. developed SegNet-based CNNdeep to predict the final infarct volume by using 9 different biomarkers as input, with an AUC of 0.88 [102]. Nishi et al. designed a 3D U-Net to extract features of DWI from LVO patients, finding that the features could be known as a clinically useful prognostic biomarker [103]. Yu et al. trained a 2.5D U-Net model using initial presentation- (baseline-) acquired magnetic resonance images (MRIs) to predict 3- to 7-day final infarct lesions without reperfusion information, with a median AUC of 0.92, proving that this method would be valuable as a starting point for fine-tuning models for specific reperfusion subgroups [104].

Lacking sufficient labeled data is one of the key challenges that has limited the progress of deep learning approaches in this domain. At present, deep learning-based models have shown great potential in a small number of datasets, making up for the lack of cumbersome processing steps of learning algorithms on a traditional machine. However, the current large-scale development of deep learning is limited by the size of the dataset, and the model has trouble of overfitting, making it difficult to exert the optimal performance of the deep learning model. Therefore, sufficient labels and model performance are key to solving the problem.

### 3.5. Deep Learning for Prediction of Imaging Functional Outcomes

Functional outcomes after acute ischemic stroke are of great concern for patients and their families, as well as physicians making clinical decisions. It can guide clinicians in advising patients and relatives about possible outcomes. The modified Rankin scale (mRS) is usually assessed within 90 days after stroke onset and has represented final clinical outcomes in several clinical trials [105]. It is often used to evaluate the prognosis of stroke and to determine the curative effect of the functional disability of patients during rehabilitation. Zero is asymptomatic and 5 is severely disabled [106].

Since 2014, lots of machine learning methods have emerged to predict the prognosis of AIS patients [28, 107]. Until 2019, there have been studies on the DL-based method predicting functional outcomes. An overview of ML-based automated algorithms for the prediction of stroke outcomes is provided in Table 5. A study developed 3 machine learning models (deep neural network, random forest, and logistic regression) and compared their predictability of predicting modified Rankin scale (mRS) score (0-2 vs. 3-6) at 90 days, with an AUC of 0.888. This study demonstrated that the use of deep learning models can accurately predict long-term outcomes and record a significantly higher AUC than the ASTRAL score [108]. Kim et al. developed an integrated modified Brunnstrom algorithm to predict the hand function and the ambulatory outcomes of a patient with corona radiata (CR) at 6 months after onset, using clinical parameters and brain magnetic resonance images as input, with an AUC of 0.891 [109]. Ding et al. employed CNNs to predict the functional outcomes at 3 months poststroke with acute brainstem infarction using clinical features, laboratory features, conventional imaging features (infarct volume and number of infarctions), and DWI neuroimaging features from 1482 patients, which achieved an extremely high AUC of 0.975 [110].

As discussed above, it can be challenging to obtain a detailed reflection of the various neurologic symptoms after ischemic stroke, such as dysarthria-clumsy hand, ataxic hemiparesis, and pure sensory stroke. In particular, there may be a discrepancy between the measured functional scores and the discomfort of the symptoms felt by the patient with these subtypes. However, a common feature of these studies is lacking sample size and external validation of DL algorithms. Future research should expand the dataset, optimize model performance, and reduce model overfitting [1, 3]. The final result is obtained through external validation of the different hospital datasets.

## 4. Outlook

Deep learning technology comes from the way the human brain works, and it is a learning process that uses deep neural networks to solve feature presentations. Compared to traditional techniques, DL has certain advantages [3]. First, the technology dramatically shortens the treatment duration. Second, it improves the satisfaction and comfort of the patients, enabling patients to enjoy the convenience brought by personalized therapeutic and precision medicine. Third, it greatly improves the work efficiency of clinicians. At present, it is widely used in various fields of medical imaging. If a deep learning-based decision support system is consistent with and correlated with individual outcomes of the patients, it has great potential to be accurate, fast, and widely accessible [4].

Rapid detection and treatment of stroke are critical to reducing morbidity and mortality. The existing application of AI in this field allows for vast opportunities to increase therapeutic options and clinical outcomes by assisting in all parts of the diagnostic and treatment settings, including detection, triage, and outcome prediction. However, deep learning still faces many challenges for stroke diagnosis. First, most analytical documents use retrospective data, and the sample size typically fluctuates from 20 to a few hundred. There is an obvious need for a larger and particularly prosperous market [5]. Second, due to the confidentiality of hospital data, most studies lack the process of external validation, resulting in low model generalization. Up-to-date, these techniques are still confined to research settings and hospitals. Future studies validating AI techniques are needed to allow for more widespread use in various practice conditions. Third, deep learning approaches still lack interpretability, and many radiologists still possess skepticism on deep learning algorithms and lack confidence in software-assisted diagnosis [7]. Currently, most attention focuses on improving the accuracy of predictions, giving AI solutions the ability to interpret their predictions that may contribute to better clinical applicability and acceptance. Using AI to identify novel disease mechanisms, as well as unrealize the links between imaging and clinical outcomes, will allow AI to accelerate the management of patients and increase safety. It can also serve as a means of hypothesis generation, paving the way for true deep learning and understanding of acute ischemic stroke.

## Figures and Tables

**Figure 1:** Applications of deep learning in acute ischemic stroke imaging analysis.

**Figure 2:** (a) CNN, (b) RNN, (c) autoencoder, (d) RBM, and (e) transformer.

**Figure 3:** The MCA territory is divided into 10 ASPECTS regions, including caudate (C), insular ribbon (I), internal capsule (IC), lentiform nucleus (L), anterior inferior frontal cortex (M1), anterior temporal cortex lateral to the insular ribbon (M2), posterior temporal cortex (M3), anterior superior frontal cortex (M4), posterior frontal cortex (M5), and parietal cortex (M6). The M4, M5, and M6 are the MCA territories superior to the M1, M2, and M3 regions, respectively.

**Table 1:** Overview of papers using deep learning techniques for early stroke diagnosis.

References	Study objective	Date published	DL-based approaches	Optimal results	Clinical implications	Limitation
Shinohara et al. [69]	Recognize acute cerebral ischemia (ACI)	2017	ANN	Precision-0.92; sensitivity-0.80; specificity-0.86	Recognition of ACI and differentiation of ACI from stroke mimics at the initial examination	Not separate patients with posterior circulation from anterior circulation stroke; not calculate precision based on stroke type or possible stroke pathogenesis; lack generalizability
Litjens et al. [67]	Identify MCA	2017	3DCNN	AUC-0.996; precision-recall AUC-0.563	Not yet at a level for routine clinical use	Small sample data sizes and lack of external validation
Lisowska et al. [68]	Identify HMCAS	2020	DCNN	Sensitivity-0.82, specifcity-0.81, and AUC-0.869	For reference and improve the accuracy of detecting HMCAS	No thin-slice CT
Cui et al. [70]	AIS diagnosis via DWI and ADC images	2021	DeepSym-3D-CNN	AUC-0.850	Early acute stroke diagnosis	Small sample data sizes

**Table 2:** Overview of documents using deep learning techniques for automated ASPECTS calculation.

References	Study objective	Date published	DL-based approaches	Optimal results	Clinical implications	Limitation
Naganuma et al. [79]	Automatic ASPECTS calculation using CT	2021	3D-BHCA	Sensitivity (0.98), specificity (0.92), and accuracy (0.97) of dichotomized ASPECTS > 5 analysis and the intraclass correlation coefficient (0.90)	Evaluation of stroke expansion to determine suitability for reperfusion therapy.	Lack external validation; old brain infarction and old brain hemorrhage disturb results; not consider reperfusion treatment.
Do et al. [41]	Automatic ASPECTS calculation using DWI	2020	RRCNN	AUC (94.1%)	Not yet at a level for routine clinical use.	Larger number of datasets should be considered to improve the performance of the model.
Cheng et al. [81]	Automatic ASPECTS calculation using DWI	2020	DCNN	ICC coefficients between interraters and between junior raters and automated scores were 0.954 and 0.923 between senior raters and automated scores were 0.939	eDWI-ASPECTS has the potential to improve standardization and provides valuable reference for less-experienced readers.	Initial description of DWI-ASPECT score is not yet clear.

**Table 3:** Overview of documents using deep learning techniques for LVO detection.

References	Study objective	Date published	DL-based approaches	Optimal results	Clinical implications	Limitation
Chatterjee et al. [88]	LVO detection	2019	CNN	Sensitivity (82%), specificity (94%), PPV (77%), and NPV (95%)	The first AI algorithm for detecting intracranial LVOs, improving EVT rates	Difficult to detect anatomic variations such as tortuosity and MCA-M2.
Shaham and R L R [89]	LVO detection	2019	RRCNN	AUC (0.914) for original brain CTA volumes, AUC (0.899) for brain tissue images	Automated detection of AIS with CTA images	Larger number of datasets should be considered to improve the performance of the model.
Yu et al. [91]	LVO detection	2020	DCNN	AUC (0.847)	Automated detection of AIS with CTA images, improving prehospital triage systems	The NCCT brain scans are thick-cut and lack prospective validation and angiogram within the acute setting.
McLouth et al. [92]	LVO detection	2021	CNNs, CINA v1.0 device (Avicenna.ai, La Ciotat, France)	Accuracy (98.1%), sensitivity (98.1%), and specificity (98.2%)	Automated detection of AIS with CTA, improving EVT rates	Not differentiate acute and nonacute LVO etiologies; not evaluate occlusions in the anterior cerebral arteries or posterior circulation.

**Table 4:** Overview of documents using deep learning techniques for evaluation of ischemic core and penumbra/prognosis.

References	Study objective	Date published	DL-based approaches	Optimal results	Imaging tool	Performance
Chen et al. [98]	Segment of stroke core lesions	2017	CNNs composed of MUSCLE Net and EDD Net	Dice score is 0.67	MR (DWI)	Comparable to manual segmentation
Ho et al. [99]	Locating stroke regions	2017	Autoencoder	AUC of 0.68	MR (PWI)	10% better than current traditional clinical method (0.58)
Sheth et al. [100]	Evaluating the volume of large vessel occlusion and determining infarct core	2017	CNN (DeepSymNet)	Determining infarct core as defined by CTP-RAPID from the CTA with AUC of 0.88 and 0.90 (ischemic core ≤ 30 mL and ≤ 50 mL)	CT (CTP)	Better than current traditional clinical method
Öman et al. [101]	Detecting AIS	2019	3D CNN	AUC of 0.93 and Dice of 0.61	CT and CTA-SI	Better than current traditional clinical method
Nielsen et al. [102]	Predicting the final infarct volume	2018	SegNet	AUC of 0.88	9 different biomarkers	—
Nishi et al. [103]	Segment of lesion and predicting clinical outcomes for LVO	2020	3D U-Net	AUC value achieved 0.81	DWI	—
Yu et al. [104]	Predicting 3- to 7-day final infarct lesions	2020	2.5D U-Net	Achieved a median AUC of 0.92	MRIs	—

**Table 5:** Overview of documents using deep learning techniques for prediction of functional outcomes.

References	Study objective	Date published	DL-based approaches	Optimal results	Imaging tool
Heo et al. [108]	Predicting mRS score	2019	Deep neural network	AUC of 0.888	MR (DWI)
Kim et al. [109]	Predicting mRS score	2020	CNN with integrated modified Brunnstrom algorithm	AUC of 0.891	Corona radiata (CR)
Ding et al. [110]	Predicting functional outcome	2021	CNNs	AUC of 0.975	Infarct volume, DWI neuroimaging features

## Data Availability

This article is a review article and the data is from Hangzhou Medical College Affiliated Lin'an District People's Hospital, Zhejiang Province.
